# Racial inequality in perinatal outcomes in two Brazilian birth cohorts

**DOI:** 10.1590/1414-431X202010120

**Published:** 2021-01-22

**Authors:** J.M. Fonseca, A.A.M. Silva, P.R.H. Rocha, R.L.F. Batista, E.B.A.F. Thomaz, F. Lamy-Filho, M.A. Barbieri, H. Bettiol

**Affiliations:** 1 Departamento de Saúde Pública, Universidade Federal do Maranhão, São Luís, MA, Brasil; 2 Departamento de Pediatria e Puericultura, Faculdade de Medicina de Ribeirão Preto, Universidade de São Paulo, Ribeirão Preto, SP, Brasil

**Keywords:** Racism, Low birth weight, Infant, Premature, Fetal growth retardation, Inequalities

## Abstract

This study aimed to estimate and compare racial inequality in low birth weight (LBW), preterm birth (PTB), and intrauterine growth restriction (IUGR) in two Brazilian birth cohorts. This was a cross-sectional study nested within two birth cohorts in Ribeirão Preto (RP) and São Luís (SL), whose mothers were interviewed from January to December 2010. In all, 7430 (RP) and 4995 (SL) mothers were interviewed. The maternal skin color was the exposure variable. Associations were adjusted for socioeconomic and biological covariates: maternal education, per capita family income, family economic classification, household head occupation, maternal age, parity, marital status, prenatal care, type of delivery, maternal pre-pregnancy BMI, hypertension, hypertension during pregnancy, and smoking during pregnancy collected from questionnaires applied at birth. Statistical analysis was done with the chi-squared test and logistic regression. In RP, newborns from mothers with black skin color had a higher risk of LBW and IUGR, even after adjusting for socioeconomic and biological variables (P<0.001). In SL, skin color was not a risk factor for LBW (P=0.859), PTB (P=0.220), and IUGR (P=0.062), before or after adjustment for socioeconomic and biological variables. The detection of racial inequality in these perinatal outcomes only in the RP cohort after adjustment for socioeconomic and biological factors may be reflecting the existence of racial discrimination in the RP society. In contrast, the greater miscegenation present in São Luís may be reflecting less racial discrimination of black and brown women in this city.

## Introduction

The concept of race is a social construction, a product of history and culture and is not restricted to a biological or genetic meaning, as traditionally understood (1). Thus, by interacting with various social position markers, race can contribute to greater or lesser exposure to different health risks (2,3).

Extensive literature from the United States highlights race as an important predictor of health outcomes. Studies show that rates of low birth weight (LBW), preterm birth (PTB), and infant mortality are higher among children born to black mothers compared to those of white mothers (4 [Bibr B05] [Bibr B06] [Bibr B07]–8). Maternal factors typically explain one-third of those black-white differences (8).

In Brazil, these data are scarce and come from studies that do not use self-classification, which is considered the most recommended procedure (2,). The “myth of racial democracy” that Brazil has reduced degrees of racial discrimination is very prevalent. Thus, the role of the racial component in generating and maintaining the very high levels of inequality in Brazilian society may be underestimated (2,10 [Bibr B11]).

Racial inequality, however, persists in Brazilian society, mainly associated with usually subtle forms of racial discrimination. Black, brown, and white people have great disparities regarding socioeconomic and demographic conditions, as well as inequalities in health indicators (12). According to a study conducted in southern Brazil, infant mortality is twice as common among black children compared to white ones (13). Regardless of birth weight, avoidable mortality rate is higher among black infants (14). According to these authors, black infants are a vulnerable racial group in Brazil.

Data from a birth cohort conducted in Pelotas, southern Brazil, showed that black infants have a higher prevalence of LBW, PTB, and intrauterine growth restriction (IUGR) (15). In Ribeirão Preto, located in the southeast of the country, the rates of LBW, PTB, and IURG births are higher for black and brown babies than for white ones, even after adjusting for socioeconomic variables. This result suggests that in addition to socioeconomic disadvantage, other factors, such as racial discrimination, may influence these health outcomes (12).

These perinatal outcomes, with emphasis on LBW and PTB, are important public health problems since they are causes of neonatal mortality in Brazil (16). In addition to race and socioeconomic characteristics, factors related to maternal age, cesarean delivery, multiple pregnancies, prenatal care, chronic gestational diseases, and maternal nutritional conditions are also directly associated with a greater risk of perinatal outcomes (17–20). In a large American study, it was observed that advanced maternal age (40 years or more) is associated with an increased risk of premature birth (17). In Brazil, data from a study conducted in the city of São Paulo showed an increased risk of low birth weight associated with maternal age and cesarean delivery (18 [Bibr B19]).

According to the National Household Sample Survey (PNAD) (21), conducted in 2015 by the Brazilian Institute of Geography and Statistics (IBGE), 45.1% of the total population (92.6 million people) reported being of brown skin color. Another 8.9% of the population (18.2 million people) declared themselves as black, and 0.8% of another color or race (indigenous or yellow). According to data from IBGE (2010), the state of Maranhão presented 76.2% of self-declared black and brown skin colors, representing one of the largest populations of black and brown people in the country (22).

Due to this large population of black and brown people, and the lack of data to clarify the factors that explain these racial inequalities in perinatal outcomes, we used data from two birth cohorts in municipalities with contrasting socioeconomic conditions (Ribeirão Preto/SP and São Luís/MA), in order to estimate and compare racial inequality in rates of LBW, PTB, and IUGR.

## Material and Methods

The data used in this research were obtained from the cohort study entitled “Etiological factors of preterm birth and consequences of perinatal factors on child health: birth cohorts in two Brazilian cities - BRISA”, developed in two municipalities with contrasting socioeconomic indicators: Ribeirão Preto/SP, located in one of the richest regions of the Southeast of the country and São Luís/MA, located in one of the most deprived regions of northeastern Brazil, from January 1st to December 31st, 2010.

Data from both cohorts are population-based. The RP birth cohort was conducted in the eight public and private maternity hospitals and hospitals with maternity services in the city, and included all hospital births of RP residents, totaling 7794 births. After excluding 42 stillbirths and 187 twins, the sample resulted in 7565 births.

In SL, the cohort included births in public and private maternity hospitals and hospitals with maternity services, which provided neonatal and childbirth care. We did not include maternity centers with less than 100 births per year. Systematic sampling was performed at each hospital, randomly selecting one in three births for an interview. After losses due to refusal or early discharge, a total of 5236 mothers living in the municipality participated in the project. Seventy stillbirths, 99 twins, and 4 cases with missing information on the mother's skin color were excluded, resulting in a sample of 5063 births.

For this research, we removed information of congenital diseases and self-reported “Asian” and “indigenous” maternal skin color information due to the small number of participants belonging to these categories, resulting in a final sample of 7430 births in RP and 4995 births in SL.

Two instruments were used to obtain the data: the mother questionnaire and the newborn questionnaire. Mothers were interviewed during the first 24 hours postpartum. During the interview, the skin color was self-reported by the mother, being categorized as white, brown, or black. The newborns had their weight measured immediately after delivery, without clothes and using electronic scales, with a precision of 5 g. According to the World Health Organization, LBW was identified when <2500 g, PTB comprised those with gestational age less than 37 weeks, and those with weight below the 10th percentile according to the Williams curve were classified as small for gestational age (SGA) (23,24). SGA was used as a proxy for IUGR.

Gestational age was calculated from the date of the last menstruation reported by the mother. The 15th day of the month was considered for cases that the day of last menstruation was unknown, but not the month. Cases of birth weight incompatible with gestational age above the 99th percentile for the reference curve were recoded as missing (23). The same procedure was used in cases of implausible gestational age (less than 20 or more than 43 weeks). In the end, a regression model imputation procedure was performed to estimate gestational age based on birth weight, parity, family income, and newborn gender.

To estimate the effect of maternal skin color on the perinatal outcomes (LBW, PTB, and IURG) and to identify possible confounders, mediators, and colliders, we developed a theoretical model (directed acyclic graph - DAG; Figure 1). The theoretical model indicated that no variable had a confounding effect on the associations between maternal skin color and perinatal outcomes.

**Figure 1:** Directed acyclic graph of the effect of maternal skin color on perinatal outcomes. The outlined green rectangle represents the exposure and the outlined blue rectangle represents the outcome. The remaining blue rectangles represent the ancestors of the outcome. The green arrows represent the causal path and the pink arrows represent the biasing path. BMI: body mass index.

The association between maternal skin color and perinatal factors was measured, and the results were analyzed using the chi-squared test, with a significance level of 0.05 through the Stata 14.0 statistical program (StataCorp, USA). Crude and adjusted odds ratios (OR) and respective 95% confidence interval (95%CI) were estimated.

The direct effect of race on perinatal outcomes was obtained by logistic regression after adjustment for the following mediators: maternal education in years of schooling (4 or less; 5 to 8; 9 to 11; 12 or more), per capita family income in minimum wages (up to 1/2; more than 1/2 to 1; more than 1 to 3; and more than 3), household head occupation (non-manual; skilled and semi-skilled manual; and unqualified or unemployed manual) (25), economic class according to the Brazilian Economic Classification Criteria of the Brazilian Association of Research Companies (26), categorized as A/B, C, D/E, with class A being the class with the highest purchasing power, maternal age (<20, 20-34, and ≥35), parity (1-4 or more), marital status (with consensual union; without consensual union), prenatal care (yes, no), type of delivery (vaginal and caesarean section), maternal pre-pregnancy BMI (underweight, normal range, overweight) (27), hypertension (yes, no), hypertension during pregnancy (yes, no), and smoking during pregnancy (yes, no).

Persistent inequality in perinatal outcomes by race (a significant direct effect) after adjustment was interpreted as possible evidence of racial discrimination. Disappearance of inequality in perinatal outcomes by race (non-significant direct effect) after adjusting implied that the effect was entirely mediated by the variables included in the models.

The research met the criteria of Resolution 196/96 of the National Health Council and its complementary norms. The project was approved by the Research Ethics Committee (CEP) of the Clinical Hospital of the Ribeirão Preto Medical School (HC-FMRP) of the University of São Paulo (USP) (Protocol No. 4116/2008) and the University Hospital of Federal University of Maranhão (HU-UFMA) (Protocol No. 4771/2008-30). All mothers signed an informed consent form.

## Results

Of the total number of mothers included in the RP analyzes, 58.9% declared themselves white, 9.7% black, and 31.4% as having brown skin color. Among the newborns, 8.2% had LBW, 13.3% were PTB, and 8.7% had IUGR. Among the mothers evaluated in SL, 18.7% had white skin color, 12.9% black skin color, and 68.4% brown skin color. Of all newborns in the city, 7.5% had LBW, 12.0% were PTB, and 10.3% had IUGR (Table 1).

**Table 1:** Perinatal outcomes in Ribeirão Preto and São Luís birth cohorts (2010).

Variables	Ribeirão Preto (n, %)	São Luís (n, %)
Low birth weight		
Yes	608 (8.2)	377 (7.5)
No	6822 (91.8)	4618 (92.5)
Preterm birth^*^		
Yes	986 (13.3)	601 (12.0)
No	6443 (86.7)	4394 (88.0)
Intrauterine growth restriction^*^		
Yes	648 (8.7)	515 (10.3)
No	6781 (91.3)	4480 (89.7)
Total	7430 (100.0)	4995 (100.0)

Total for Ribeirão Preto may not reach 7430 observations due to missing data.

In the RP birth cohort, the percentage of LBW was significantly higher among children born to mothers with black skin color (11.8%) compared to children born to mothers with brown (8.9%) or white skin color (7.2%) (P<0.001). The percentage of IUGR was higher among children born to mothers with black skin color (13.2%) compared to children born to mothers with brown (9.2%) or white skin color (7.7%) (P<0.001). The percentage of PTB showed no difference between children born to mothers with different skin colors (P=0.115) (Table 2). Among SL births, there was no difference between the proportions of births with LBW (P=0.859), PTB (P=0.220), and IUGR (P=0.062) between the different groups of maternal skin color (Table 3).

**Table 2:** Perinatal, socioeconomic, and biological variables according to maternal skin color in the Ribeirão Preto birth cohort, 2010.

Variables	Skin color			P value
	White (n, %)	Brown (n, %)	Black (n, %)	
Low birth weight				<0.001
Yes	315 (7.2)	208 (8.9)	85 (11.8)	
No	4064 (92.8)	2125 (91.1)	633 (88.2)	
Preterm birth				0.115
Yes	556 (12.7)	320 (13.7)	110 (15.3)	
No	3823 (87.3)	2013 (86.3)	607 (84.7)	
Intrauterine growth restriction				<0.001
Yes	339 (7.7)	214 (9.2)	95 (13.2)	
No	4040 (92.3)	2118 (90.8)	623 (86.8)	
Maternal education (years)				<0.001
≥12	3166 (72.3)	1025 (43.9)	338 (47.1)	
9-11	466 (10.7)	390 (16.7)	114 (15.9)	
5-8	649 (14.8)	746 (32.0)	209 (29.1)	
≤4	91 (2.1)	172 (7.4)	57 (7.9)	
Missing	7 (0.2)	0 (0.0)	0 (0.0)	
Per capita family income (minimum wages)				<0.001
>3	723 (16.5)	78 (3.3)	15 (2.1)	
>1-3	1655 (37.8)	680 (29.1)	215 (29.9)	
>1/2-1	880 (20.1)	769 (33.0)	212 (29.5)	
≤1/2	365 (8.3)	434 (18.6)	176 (24.5)	
Missing	756 (17.3)	372 (15.9)	100 (13.9)	
Family economic classification				<0.001
A/B	2449 (55.9)	630 (27.0)	161 (22.4)	
C	1487 (34.0)	1172 (50.2)	381 (53.1)	
D/E	202 (4.6)	359 (15.4)	126 (17.6)	
Missing	241 (5.5)	172 (7.4)	50 (6.9)	
Household head occupation				<0.001
Non-manual	1214 (27.7)	256 (11.0)	48 (6.7)	
Skilled/semiskilled manual	1935 (44.2)	1114 (47.8)	321 (44.7)	
Unqualified manual/unemployed	690 (15.8)	711 (30.4)	238 (33.1)	
Missing	540 (12.3)	252 (10.8)	111 (15.5)	
Maternal age				<0.001
<20	444 (10.1)	381 (16.3)	116 (16.2)	
20-34	3301 (75.4)	1722 (73.8)	534 (74.4)	
≥35	634 (14.5)	230 (9.9)	68 (9.5)	
Parity				<0.001
1	2030 (46.4)	943 (40.4)	287 (40.0)	
2	1347 (30.8)	633 (27.1)	196 (27.3)	
3	583 (13.3)	406 (17.4)	105 (14.6)	
≥4	419 (9.6)	351 (15.1	130 (19.1)	
Marital status				<0.001
With consensual union	3892 (88.9)	1973 (84.6)	560 (78.0)	
Without consensual union	481 (11.0)	359 (15.4)	158 (22.0)	
Missing	6 (0.1)	1 (0.1)	0 (0.0)	
Prenatal care				<0.001
Yes	4345 (99.2)	2290 (98.2)	695 (96.8)	
No	28 (0.6)	43 (1.8)	23 (3.2)	
Missing	6 (0.1)	0 (0.0)	0 (0.0)	
Type of delivery				<0.001
Vaginal	1387 (31.6)	1261 (54.1)	413 (57.5)	
Cesarean section	2991 (68.3)	1072 (45.9)	305 (42.5)	
Missing	1 (0.1)	0 (0.0)	0 (0.0)	
Maternal pre-pregnancy BMI				<0.001
Underweight	268 (6.1)	161 (6.9)	46 (6.4)	
Normal range	2198 (50.2)	1010 (43.3)	278 (38.7)	
Overweight	864 (19.7)	467 (20.0)	136 (18.9)	
Obese	465 (10.6)	227 (9.7)	85 (11.8)	
Missing	584 (13.3)	468 (20.1)	173 (24.1)	
Hypertension				0.029
Yes	104 (2.4)	68 (2.9)	29 (4.0)	
No	4258 (97.2)	2260 (96.9)	684 (95.3)	
Missing	17 (0.4)	5 (0.2)	5 (0.7)	
Hypertension during pregnancy				<0.001
Yes	479 (10.9)	311 (13.3)	126 (17.6)	
No	3882 (88.7)	2015 (86.4)	588 (81.9)	
Missing	18 (0.4)	7 (0.3)	4 (0.6)	
Smoking during pregnancy				<0.001
Yes	412 (9.4)	325 (13.9)	130 (18.1)	
No	384 (8.8)	178 (7.6)	53 (7.4)	
Missing	3583 (81.8)	1830 (78.5)	535 (74.5)	
Total	4379 (100.0)	2333 (100.0)	718 (100.0)	

BMI: body mass index. Chi-squared test.

**Table 3:** Perinatal, socioeconomic, and biological variables according to maternal skin color in the São Luís birth cohort, 2010.

Variables	Skin color			P value
	White (n, %)	Brown (n, %)	Black (n, %)	
Low birth weight				0.859
Yes	67 (7.2)	259 (7.6)	51 (7.9)	
No	865 (92.8)	3160 (92.4)	593 (92.1)	
Preterm birth				0.220
Yes	97 (10.4)	421 (12.3)	83 (12.3)	
No	835 (89.6)	2998 (87.7)	561 (87.1)	
Intrauterine growth restriction				0.062
Yes	81 (8.7)	376 (11.0)	58 (9.0)	
No	851 (91.3)	3043 (89.0)	586 (91.0)	
Maternal education (years)				<0.001
≥12	285 (30.6)	374 (10.9)	86 (13.4)	
9-11	477 (51.2)	2033 (59.5)	380 (59.0)	
5-8	147 (15.8)	840 (24.6)	134 (20.8)	
≤4	22 (2.3)	160 (4.7)	44 (6.8)	
Missing	1 (0.1)	12 (0.3)	0 (0.0)	
Per capita family income (minimum wages)				<0.001
>3	146 (15.7)	136 (3.9)	25 (3.9)	
>1-3	244 (26.2)	525 (15.4)	116 (18.0)	
>1/2-1	200 (21.5)	857 (25.1)	153 (23.8)	
≤1/2	208 (22.3)	1237 (36.2)	249 (38.7)	
Missing	134 (14.4)	664 (19.4)	101 (15.7)	
Family economic classification				<0.001
A/B	333 (35.7)	475 (13.9)	86 (13.4)	
C	431 (46.2)	1751 (51.2)	342 (53.1)	
D/E	135 (14.5)	963 (28.2)	181 (28.1)	
Missing	33 (3.5)	230 (6.7)	35 (5.4)	
Household head occupation				<0.001
Non manual	304 (32.6)	594 (17.4)	120 (18.3)	
Skilled/semiskilled manual	332 (35.2)	1468 (42.9)	230 (35.7)	
Unqualified manual/unemployed	264 (28.4)	1240 (36.3)	279 (43.3)	
Missing	32 (3.4)	117 (3.4)	15 (2.3)	
Maternal age				<0.001
<20	138 (14.8)	703 (20.6)	93 (14.4)	
20-34	701 (75.2)	2495 (72.9)	485 (75.3)	
≥35	93 (10.0)	221 (6.5)	66 (10.3)	
Parity				<0.001
1	409 (43.9)	1359 (39.7)	261 (40.5)	
2	284 (30.5)	970 (28.4)	181 (28.1)	
3	138 (14.8)	581 (17.0)	86 (13.4)	
≥4	101 (10.8)	509 (14.9)	116 (18.0)	
Marital status				<0.001
With consensual union	798 (85.6)	2746 (80.3)	497 (77.2)	
Without consensual union	134 (14.4)	673 (19.7)	147 (22.8)	
Prenatal care				<0.001
Yes	923 (99.0)	3352 (98.0)	621 (96.4)	
No	9 (1.0)	67 (2.2)	23 (3.6)	
Type of delivery				<0.001
Vaginal	349 (37.4)	1956 (57.2)	358 (55.6)	
Cesarean section	583 (62.6)	1463 (42.8)	286 (44.4)	
Maternal pre-pregnancy BMI				<0.001
Underweight	72 (7.7)	323 (9.5)	61 (9.5)	
Normal range	503 (54.0)	1563 (45.7)	255 (39.6)	
Overweight	119 (12.8)	392 (11.5)	93 (14.4)	
Obese	35 (3.7)	114 (3.3)	37 (5.8)	
Missing	203 (21.8)	1027 (30.0)	198 (30.7)	
Hypertension				0.968
Yes	30 (3.2)	119 (3.5)	24 (3.7)	
No	901 (96.7)	3297 (96.4)	619 (96.1)	
Missing	1 (0.1)	3 (0.1)	1 (0.2)	
Hypertension during pregnancy				0.213
Yes	153 (16.4)	538 (15.7)	124 (19.3)	
No	779 (83.6)	2879 (84.2)	520 (80.7)	
Missing	0 (0.0)	2 (0.1)	0 (0.0)	
Smoking during pregnancy				0.103
Yes	27 (2.9)	141 (4.1)	34 (5.3)	
No	67 (7.2)	262 (7.7)	39 (6.1)	
Missing	838 (89.9)	3016 (88.2)	571 (88.6)	
Total	932 (100.0)	3419 (100.0)	644 (100.0)	

BMI: body mass index. Chi-squared test.

Low education (≤4 years of schooling) was approximately four times higher among black (7.9%) and brown (7.4%) mothers than among white ones (2.1%) in RP (P<0.001) (Table 2). Similarly, low education was approximately double among brown mothers (4.7%) and almost triple among black mothers (6.8%) compared to white (2.3%) and brown mothers in SL (P<0.001) (Table 3).

Per capita family income, family economic classification, and household head occupation also showed statistically significant differences according to maternal skin color in the two cities (Tables 2 and 3). In RP and SL, white mothers had a per capita family income of more than three minimum wages (16.5% in RP, 15.7% in SL) higher than brown (3.3% in RP, 3.9% in SL) and black (2.1% in RP, 3.9% in SL) (P<0.001) mothers.

In addition, the percentage of participants in classes D and E was almost four times higher among black mothers (17.6%) compared to white ones (4.6%) (P<0.001) among RP residents. In SL, the percentage in these categories among the brown (28.2%) and black (28.1%) mothers were practically double that of white (14.5%) mothers (P<0.001). Heads of households of black mothers in RP (33.2%) had a two times higher percentage of unqualified or unemployed occupations compared to those of families of white mothers (15.8%) (P<0.001). This difference was 1.5 times higher in SL (P<0.001) (Tables 2 and 3).

Mothers with black and brown skin colors had a higher percentage of non-consensual union (P<0.001), lower percentage of cesarean section (P<0.001), higher percentage of mothers with more than four children (P<0.001), and higher percentage of mothers without prenatal care compared to white mothers in the two cities. In RP and SL, the percentage of mothers within normal range in maternal pre-pregnancy BMI was higher for white mothers (50.2% in RP, 54% in SL) than brown (43.3% in RP, 45.7% in SL), and black mothers (38.7% in RP, 39.6% in SL) (P<0.001) (Tables 2 and 3). In RP, brown and black mothers were younger and, similarly, brown mothers were younger in SL (P<0.001) (Tables 2 and 3).

In the two cities, there was no significant difference between mothers with different skin color regarding hypertension (P=0.029 - RP; P=0.968 - SL), however, in RP, a higher percentage of black mothers had hypertension during pregnancy compared to white mothers (P<0.001) (Tables 2 and 3). Only in RP, smoking during pregnancy was significantly higher among children born to black mothers (18.1%) compared to children born to mothers with brown (13.9%) or white skin color (9.4%) (P<0.001) (Table 2).

In RP, after adjusting for maternal education, per capita family income, family economic classification, household head occupation, maternal age, parity, marital status, prenatal care, type of delivery, maternal pre-pregnancy BMI, hypertension, hypertension during pregnancy, and smoking during pregnancy, only black skin color remained independently associated with LBW and IUGR. In the SL cohort, maternal skin color was not associated with LBW, PTB, and IUGR after adjustment for socioeconomic and biological variables (P>0.05) (Supplementary Table S1).

## Discussion

Black and brown mothers had more unfavorable socioeconomic indicators and biological variables compared to white mothers in both cohorts. Children born to black mothers had a higher risk of LBW and IUGR and the direct effect of race on perinatal outcomes persisted in RP after adjusting for socioeconomic and biological factors. In SL, however, maternal skin color was not associated with a higher risk of LBW, PTB, and IUGR.

According to a literature search, this is the first study that aimed to evaluate and compare two population-based Brazilian birth cohorts in regions with contrasting socioeconomic characteristics concerning racial inequalities. A strong point of the present study is that perinatal data were collected in the first hours after delivery, reducing the likelihood of memory bias. Also, the self-classification of race by mothers can also be considered a strong point of the research, since this is the most recommended procedure to be used (9,10). However, gestational age was estimated from the date of the last menstruation reported by the mother. Missing data on gestational age was imputed in a regression model based on birth weight, parity, family income, and gender of the newborn to reduce bias due to the exclusion of missing cases. Also, information on mothers’ drug addiction was not obtained.

In both cohorts, white mothers showed a clear advantage compared to those of black and brown skin color in relation to schooling. These data corroborate previous studies that showed that black and brown people have less access to education than white people. According to IBGE census data (2010), the percentage of illiterate people is almost three times higher among black (14.4%) and brown individuals (13.0%), compared to those of white skin color (5.9%). As in the study by Barros et al. (15), with data from a Pelotas birth cohort, there was a clear socioeconomic disadvantage of black mothers compared to white mothers. In the present study, black and brown mothers from both cohorts had lower family per capita income, a higher percentage belonged to the less favored economic classes and had heads of households in the unqualified and unemployed manual category compared to white mothers. Thus, black and brown skin colors are still associated with unfavorable socioeconomic conditions, presenting a racial bias.

According to data from the Institute of Applied Economic Research (2011), among the richest 10%, the proportion of the black population was approximately 24% in 2009, much lower than the white population. In assessing the first tenth of the distribution (the poorest 10% of the population), black people accounted for 72% (28). This fact shows that although Brazil is considered a country in which the myth of racial democracy prevails, racial inequality is still present and has considerable influence on socioeconomic conditions.

In the RP cohort, brown and black mothers were younger and fewer were in consensual union, corroborating the findings by Silva et al. (12), who analyzed a birth cohort in the same city in the years 1978/79. Those authors showed that brown and black mothers presented higher percentages of pregnancy during adolescence and absence of a companion than white women, suggesting that unplanned pregnancy is more frequent among non-white women.

In both cohorts, brown and black mothers had more vaginal delivery compared to white mothers, corroborating the findings by Silva et al. (12) and Barros et al. (15). This result can be considered a positive indicator, since these mothers would have a lower risk of unnecessary cesarean deliveries. In a study by Moreira et al. (18), cesarean delivery was associated with the occurrence of low birth weight (25).

Silva et al. (12) observed that the rates of LBW and IUGR were lower among white individuals compared to black and brown individuals. The results of the present study corroborate the findings of that study, in which children born to black mothers were at higher risk for these perinatal outcomes even after adjusting for socioeconomic variables, suggesting an unlikely genetic explanation or the presence of racial discrimination to explain this difference.

The PTB rate in the RP cohort of the present study, however, did not differ between newborns of white, brown, and black mothers, contradicting other studies. Oliveira et al. (29), in a systematic review with meta-analysis of articles published from 2010 to 2014, observed that black women are 1.5 times more likely to have PTB compared to non-black women. A possible explanation for not detecting the association is that there is really no difference in preterm birth rates between black and brown compared to white mothers in RP.

In contrast, in the SL cohort, the rates of LBW, PTB, and IUGR were not different from newborns of white, brown, and black mothers. These results led to the conclusion that maternal skin color was not a risk factor for perinatal outcomes in SL, even with the existence of socioeconomic and biological inequalities between different races.

The conflicting results between the two cohorts may reflect the greater racial discrimination in the city of Ribeirão Preto, in the southeast of the country, that may be due to the lower number of black (9.7%) and brown (31.4%) mothers in this locality, compared to the city of São Luís, in the Brazilian Northeast, where black mothers account for 12.9% and brown mothers represent 68.4%; other factors not assessed in this study might also account for the difference. Mehra et al. (8) found that differences in perinatal outcomes between black and white populations are higher in segregated areas and lower in non-segregated areas. Thus, the greater miscegenation present in the city of São Luís could be leading to a reduction in inequality between individuals with different skin colors, perhaps resulting in less racial discrimination.

## Supplementary Material

Click here to view [pdf].
